# Nursing Progress of Hypertonic Saline Inhalation in the Treatment of Infantile Bronchitis Based on Image Enhancement

This article has been retracted.

**DOI:** 10.1155/2022/5092969

**Published:** 2022-01-22

**Authors:** Haiyan Li, Yangang Song, Xue Chen, Hesheng Sun

**Affiliations:** Sunshine Union Hospital, Shandong Province 261000, China

## Abstract

The onset of bronchiolitis is closely related to the anatomical characteristics of the bronchi in children of this age. This kind of injury is caused by epithelial necrosis, nasal mucosa, and mucosal edema caused by narrowing and blockage of the trachea. Children with this serious phenomenon will have respiratory and heart failure, which threatens the life of children to a large extent. In this paper, based on image enhancement technology, hypertonic saline aerosol inhalation treatment of pediatric bronchiolitis nursing care, through related cases, the application of image enhancement technology in hypertonic saline aerosol inhalation therapy and pediatric bronchiolitis is analyzed, and the tone mapping function is used. Tone mapping functions, hereditary arithmetics, and slope regimes for experimental field capture and detection were used for the objective of therapeutic approaches for the treatment of pediatric capillary pneumonia by hypertonic inhalation. Experimental results show that imaging technology hypertonic inhalation can control the main symptoms of bronchiolitis in infants and young children. Inhalation of 3% saline can shorten the course of moderately chronic children to half a year and can reduce the length of hospital stay by a quarter of the original requires hospitalization time, and the cure rate of pediatric bronchiolitis is increased to 93.7%.

## 1. Introduction

In recent years, we have tried automatic interferon therapy, as interferon is a more commonly used drug for allergic bronchitis in clinical use, and interferon nebulized inhalation can be used for symptomatic treatment if relevant symptoms of the disease occur. Which has a therapeutic effect on this disease and asthma. Nebulized aspiration therapy is based on the nebulized particles being small and homogenous in size, which can easily enter and deposit directly into the tiny bronchial tubes, thus, enhancing the benefits of rapid and high effective drug administration [1]. Its antiviral and immune regulation of the body exerts its effects by inducing cells of the body to produce a broad-spectrum antiviral protein. Medical imaging is an important source and information source of modern medical appraisal. With the advanced application of medical imaging technology in the medical process, the accuracy and timing of medical examination have also been greatly improved [2]. For example, ultrasound and X-ray examinations, some scholars have shown that the diagnostic accuracy rate under medical imaging tests is over 97%. Capillary bronchitis is only seen before the age of 2 years and is mainly caused by syncytial virus infection of the lower respiratory tract, which is manifested by a “whirring” wheezing sound after a cold in children under 2 years of age or a croup sound on the doctor's stethoscope. The syncytial virus stimulates the immune response to secrete large amounts of mucus, which affects the respiratory function of the respiratory system, resulting in respiratory symptoms in infants and children. In addition, immunodeficiency caused by infection is also the key to disease development [3]. It has been found that the main target of immune imbalance is T-lymphocytes, and it has been shown that the absence of T-lymphocytes leads to immune dysregulation and wheezing.

In recent years, pulmonary embolism detection technology has been applied to the diagnosis and diagnosis of respiratory diseases in infants and children, and the lung function indicators obtained by this technology can be used as golden indicators to monitor the lung function status of asthma patients. The lung sounds during respiration are recorded, and these vibration signals are recorded and analyzed by imaging and quantification using sensors. The signal processing technology can be used to realize dynamic imaging with the help of computers, so that the function and structure of the airway can be reflected visually, and the changes in airway function can be understood through signal analysis. Although there are many drugs available for the treatment of bronchiolitis in children, there is currently no effective treatment for bronchiolitis in children to cure bronchitis in children, and there are currently immunotherapy methods. Mucus inflammatory secretions and necrotic cells in the lumen form phlegm thrombi, partial or complete obstruction of the respiratory system leads to severe obstructive atelectasis or emphysema, causing respiratory insufficiency [4]. By reading references on pediatric capillary bronchiectasis, it was found that the researches indicated that 17-60% of children with capillary Bronchiectasis are likely to have recurrence in the further future [5]. In addition, the early onset and rapid progress of bronchiolitis pose a major threat to the lives and health of children and adolescents. Since the increase in the quantity of children with bronchitis has significantly affected the children themselves, their families, and society as a large number, it is imperative to minimize the prevalence of asthma by promoting bronchitis prevention.

Domestic research on the treatment of bronchiolitis by hypertonic inhalation is most limited to one of the drugs, or the therapeutic effect of one of the drugs and other types of drugs. There are few studies on bronchitis, and its medical effects are worth exploring. The remaining stages of Reju's work aim to end the optimization of scores used in the fractional filtering of image enhancement techniques in digital image processing. The work is done on the MATLAB platform. This work first compares and studies fractional-order filters and integer-order kernel filters (such as Sobel and Prewitt filters) for edge detection and boundary detection of various digital images. Considering the application of fractional filtering in medical images, this work is done by using magnetic resonance imaging (MRI). Analyze the noise performance of these filters after adding random Gaussian noise. The mean square error (MSE) and peak signal-to-noise ratio (PSNR) of the detected images are used as evaluation methods for comparison. This project demonstrates a visual comparison of filtering capabilities in medical image enhancement. It has been proved that the fractional filter is better than the integer-order filter [6]. With the established role in cystic fibrosis and bronchiectasis, nebulized antibiotics are increasingly used to treat respiratory infections in critically invasive, mechanically ventilated adult patients. Although the evidence describing its effectiveness and safety is limited, in an era where new strategies are needed to improve the effectiveness of antibiotics due to the shortage of new drugs and the increase in antibiotic resistance, the potential of nebulizing antibiotics to optimize treatment is considered to be of high concern. Especially in patients infected with multidrug resistance (MDR) pathogens. This position paper of the European Society of Clinical Microbiology and Infectious Diseases is based on systematic reviews and meta-analysis. RelloJ provides recommendations on the use of nebulized antibiotics in invasive mechanically ventilated adults based on the recommended grading evaluation, development, and evaluation (GRADE) method. Case characteristics two children (a 1-year-old girl and a 7-year-old boy) had recurrent respiratory distress and acute exacerbations. Bronchoscopy showed a membrane-like cast. In addition to asthma treatment, the two children also received nebulized N-acetylcysteine treatment. The results were asymptomatic, and there was no recurrence after 9 months of follow-up. News nebulized N-acetylcysteine may help prevent the recurrence of plastic bronchitis caused by asthma [7]. These researches on medical image enhancement technology, atomization therapy, etc. have a certain reference value. However, according to careful study, most of these studies are focused on a single field. The combination of the two makes the two more important. Well-integrated research is still lacking in both literature and examples.

The research in this paper is based on the effective implementation of image contrast enhancement by image enhancement technology. A study of the therapeutic modality of hypertonic saline nebulized inhalation was conducted to establish an experiment in pediatric capillary bronchitis care based on this premise. In this study, an optimized speed optimization algorithm based on genetic algorithm is used to process the image brightness in combination with retinex process to remove halos and finally restore high level of color images to overcome color inconsistency and problems such as multidimensional display size migration. The analysis of the method of information loss and blur caused by noncritical information and the relationship between adjacent pixels reveals a two-angle transition and enhancement method for optical vision. Infrared imaging depends on image display quality evaluation and imaging information design density, and the application of genetic algorithms and the study of image enhancement skills unfold a pioneering new approach to fog therapy experiments for the treatment of pediatric capillary bronchitis conditions.

## 2. Nursing Progress of Bronchiolitis

### 2.1. Infantile Bronchiolitis

With the increasing incidence of tracheobronchial tuberculosis, tracheobronchial tuberculosis has become the leading cause of benign respiratory stenosis in my country [8]. Bronchiolitis is a very common lower respiratory disease, with a high incidence in infants and children mainly bronchiolopathy. An important function is nasal congestion, also called respiratory pneumonia, which is a major lung disease. The most common age of onset of bronchiolitis is less than two years, especially between two months and six months [9]. As a result of the special respiratory tissue configuration of babies and children, the disease is characterized by significant symptoms of respiratory obstruction, rapid evolution of the disease. The clinical manifestation of infantile bronchiolitis is a viral upper respiratory tract infection. Entering the lower respiratory tract after a few days, manifested as persistent cough, tachypnea, and increased work of breathing.

Inflammatory substances can cause tracheal smooth muscle spasm and contraction, vasodilation, and plasma leakage. The development of the glands increases the narrowing and blockage of the abdominal lumen with accompanying respiratory and functional impairment. The main manifestations are wheezing and wheezing in the lungs. At the same time, there is also paroxysmal dyspnea. Because the lesion is located in the lower respiratory tract, the symptoms of lower respiratory tract obstruction are the main symptoms, which are dyspnea and wheezing in the lungs. When the virus infection accumulates the airway epithelium, and the airway inflammation gradually invades the bronchi and alveoli, wheezing is prone to increase, which further forms the body's ventilation and ventilation dysfunction. The respiratory mucosal edema and airway epithelial cell necrosis can cause partial or total obstruction of the airway in severe cases, and hypoventilation can lead to rapid breathing, hypoxemia, and even respiratory failure [10]. Since overclogging will cause an increase in unwanted fluid drainage and a decrease in fluid retention in the system, this will lead to dryness of the upper airways and difficulty in discharge of airway secretions.

### 2.2. Image Enhancement Technology

Image enhancement refers to presenting the local information of interest in the image, deleting or removing other information, analyzing the image, and preidentifying different identities for different applications in order to meet the needs of specific applications [11]. The original image information is a set of methods for device identification better for people. Modern medicine is a reliable source of information provided by medical imaging, and this is because military video often has a significant role in the diagnosis of diseases, therapy programs, and the choices of treatment methods and approaches. Wavelength shift-based advanced imaging intensification algorithms were researched to optimize the low-resolution X-ray image enhancement [12]. Use special conditions to select the wavelength base, and then adaptively filter the links in all directions after the waveform changes to obtain the required rich text links. How to use advanced algorithms to process and capture medical images with prominent information to meet specific needs, and obtain high-definition, information-rich medical images with high exposure sharing ratio and high noise is important for doctors' examinations, the improvement of the medical field, and the improvement of patient conditions significance.

Considering that the vision is more sensitive to perceive the gray level change of the central gray area of the image than the high and low gray areas, in order to avoid the blurring of the image during the review process, the contrast area of the image is used to distinguish the image altar area from the edge information area. And the strength of this use can be obtained with more fine details and more accentuated density of the noise ratio, which can be of great advantage for the purpose of evaluation and as a result of further processing of medical images [13]. The research on image enhancement technology in this paper mainly includes the enhancement of color image itself, the enhancement of multidisplay image compression based on image field, and the enhancement of multi-image compression based on frequency range. The image domain enhancement method is generally expressed as

(1) $$\begin{array}{c} h\left(a,b\right)=S\left[O\left(a,b\right)\right]\oint \frac{n_{k}}{n}. \end{array}$$

*O* (*a*, *b*) is the image to be enhanced, *h*(*a*, *b*) is the image after enhancement, *S* represents the area enhancement function, and the relationship between pixel and frequency is *n*_*k*_/*n*. It can be obtained after processing the image signal using probability theory:

(2) $$\begin{array}{c} h\left(a,b\right)=S^{-1}\left[G\left(u,v\right)*s\left(u,v\right)\right]\int_{v}^{u}⊗\left|\frac{d_{b}}{d_{a}}\right|, \end{array}$$

(3) $$\begin{array}{c} T\left(a,b\right)=\int_{b}^{a}h_{u,v}\left(\overset{1}{\underset{i=1}{\sum }}\frac{n_{k}}{n}\right). \end{array}$$

The calculation of *T*(*a*, *b*) results in the value of the change function of image equalization, *G*(*u*, *v*) denotes the grayscale frequency of the image, and the product of the frequency range *s*(*u*, *v*) of the image can represent the previous region enhancement function [14]. The first step of which is the degree of gray area of the image is |*d*_*b*_/*d*_*a*_|, and the degree of darkness of the gray area of the image is ∫_*a*_^*b*^*h*_*u*,*v*_. If the gray areas of the image are evenly distributed, there are

(4) $$\begin{array}{c} \text{Average}=\Omega f_{\min}^{a}+\left(f_{\max}-f_{\min}\right)•n_{\left(u,v\right)}\underset{a<b}{\sum }\left(u,v\right). \end{array}$$

The gray level transformation range is

(5) $$\begin{array}{c} h\left(m,n\right)=\frac{\left(M,N\right)\left[F\left(u,v\right)-b\right]}{a-b}+n, \end{array}$$

(6) $$\begin{array}{c} f\left(m,n\right)=n^{k\left|f\left(m,n\right)-v\right|}-1. \end{array}$$

In formula (5), *h* (*m*, *n*) is the range before transformation, and the output image is (*M*, *N*); the linear gray scale transformation is determined by *n*^*k*^. When 0 < *M* − *N*/*a* − *b* < 1, in the control of the inhalation volume and the continuity of drug molecules, etc., the probability theory of the image signal is used to control the image rendering grayscale range will be compressed, so that the originally bright parts will turn dark. On the contrary, when *M* − *N*/*a* − *b* > 1 is original dark part will become brighter due to expansion.

Processing according to genetic algorithm [15]:

(7) $$\begin{array}{c} \left\{\begin{array}{c} \mathrm{Min}\langle g_{1}=f_{1}\left(x\right),g_{2}=f_{2}\left(x\right),\cdots ,g_{n}=f_{n}\left(x\right)\rangle ,\\ p.d.\left[f_{n}\left(x0\leq 0\right.,n\in \left(1,x\right)\right], \end{array}\right. \end{array}$$

(8) $$\begin{array}{c} \langle \begin{array}{c} a^{n}=100•\left[u\left(\frac{x^{-1}}{x}\right)-u\left(\frac{x}{x_{-1}}\right)\right],\\ b^{m}=40*\left[v\left(\frac{y^{-1}}{y}\right)-v\left(\frac{y}{y_{-1}}\right)\right]. \end{array} \end{array}$$

*a* ^*n*^ is the color information, and *x*^−1^/*x*, *x*/*x*_−1_ is the reference white point value. The mathematical expression of the contrast before and after the dark color range transformation of the image is

(9) $$\begin{array}{c} h^{\prime }\left(a,b\right)=\frac{z}{l_{\max}-l_{\min}}\times \left(l\left(a,b\right)-l_{\min}\right)+l_{0}. \end{array}$$

The general expression of logarithmic transformation is

(10) $$\begin{array}{c} p\left(a,b\right)=Q•\delta \left[1+h\left(a,b\right)-\min_{a}^{b}\right]. \end{array}$$

The minimum gray value of the input image after logarithmic transformation is min_*a*_^*b*^. Its gradient magnitude is expressed as

(11) $$\begin{array}{c} K\left[f\left(a,b\right)\right]=\left[\begin{array}{c} \frac{\lambda f}{\lambda a}\\ \frac{\varepsilon f}{\varepsilon b} \end{array}\right], \end{array}$$

(12) $$\begin{array}{c} {\left|K\left[f\left(a,b\right)\right]=\left\{\left[f\left(a,b\right)-f\left(a-1,b\right)\right]\right\}\right|}^{2}+{\left[f\left(a,b\right)-f\left(a,b+1\right)\right]}^{1/2}. \end{array}$$

The calculation of the gradient value is mainly due to the difference between the edge area of the image and the flat area and the detail area.

The image enhancement technique in this paper is the histogram grayscale transform, the differential enhancement method mentioned in the references to optimize the parameters, and the experiments show that for fractional order differentiation in appropriate cases can achieve the increase of high frequencies to preserve low frequencies. While integer-order differentiation is not achievable, its performance is higher than integer-order differentiation. However, histogram equalization can achieve global contrast enhancement for the overall darker and brighter images with low contrast. Therefore, this paper chooses grayscale transform as the main method for image enhancement, as shown in Figure 1.

### 2.3. Hypertonic Saline Inhalation Therapy

In recent years, aerosol inhalation has been widely used in the treatment of infantile wheezing diseases. Because the children are younger and have poor medication compliance, their liver function is still underdeveloped. This method of administration is simple. It is easy to do, with small side effects, and can quickly let the medicine reach the bronchial lesions, and the effect is rapid. Therefore, the treatment of bronchiolitis is also inseparable from atomized inhalation, and there are many types of drugs used in atomized inhalation treatment [16]. For the treatment of bronchiolitis in infants and children, in addition to inhaled receptor agonists and glucocorticoids, fluid supplementation, and nutritional support therapy, in children with acute to severe cases of chronic to multiple sclerosis, respiratory management support can be useful in reducing pediatric clinical problems and facilitating physical rehabilitation. Foreign scholars have conducted clinical trials on more than 400 children with bronchiolitis. Among them, 85% of the children only use 3% hypertonic saline for nebulization and do not use combined bronchodilator therapy [17]. Another 15% of the children were treated with 3% hypertonic saline combined with bronchodilator nebulization, and the aggravation of cough and asthma symptoms was observed 3 days after drug withdrawal. The child was sprayed with 3% hypertonic saline combined with bronchodilator and observed the worsening of cough and asthma symptoms 3 days after stopping the drug. The results showed that 3% hypertonic saline is safe in clinical treatment. This study shows that hypertonic saline has a positive effect in the treatment of bronchiolitis, is safe and convenient, simple, and easy to operate, and is worthy of promotion, especially in basic hospitals and community medical institutions without aerosol inhalation conditions. It has more important promotion value and significance [18].

As a representative of inhalation therapy, atomization therapy has mature technical support and affirmative therapeutic effect [19]. As a rehabilitation device for the treatment of respiratory diseases, medical nebulizers have long been transferred from the professional medical industry to the family. If the atomization process is regarded as a wavelet function, it can be expressed as

(13) $$\begin{array}{c} T_{\psi }=\overset{+\alpha }{\underset{-\alpha }{\sum }}\frac{{\left|\overset{\cdot }{\psi \left(r\right)}\right|}^{2}}{\left|r\right|}ur<\beta . \end{array}$$

The calculated result is a linear equation for the formation of atomized particles. A group of connected atomized particles can be composed [20]:

(14) $$\begin{array}{c} \psi_{x,y}\left(e\right)=\frac{1}{\sqrt{x}}\psi \left(\frac{e-b}{x}\right)x,y\notin e. \end{array}$$

The continuous linear wave mother can be expressed as

(15) $$\begin{array}{c} G_{i}\left(x,y\right)=x,\psi_{x,y}⊗\frac{1}{\sqrt{b}}\int f\left(\psi •\frac{y-b}{a}\right), \end{array}$$

(16) $$\begin{array}{c} x\left(e\right)=\frac{1}{h_{e}}\int_{-\varepsilon }^{+\varepsilon }\int_{-\alpha }^{+\alpha }\psi_{x,y}\frac{exey}{x^{2}}. \end{array}$$

This calculation method is convenient to transform the wavelet function into a two-dimensional space and perform the inverse transformation into the original function in the space domain [21]. The inverse transformation can be expressed as

(17) $$\begin{array}{c} \psi_{a.b}\left(x,y\right)=\frac{1}{\sqrt{e}}\psi \left(\frac{b-a}{x},\frac{a-b}{y}\right)\int_{-\alpha }^{\alpha }. \end{array}$$

After performing the inverse transformation, a certain atomized particle is formulated as (*m*, *n*), and the corresponding wavelet mother function:

(18) $$\begin{array}{c} \lambda_{m,n}\left(e\right)=a_{1}^{-m/2}\psi {\left(\frac{a-{nb}_{o}a_{0}}{a_{0}^{m}}\right)}^{n}, \end{array}$$

(19) $$\begin{array}{c} \lambda_{m,n}\left(e\right)=2^{m/2}\psi \left(2^{-m}y-n\right)\varepsilon . \end{array}$$

In formula (17), when *a*_0_ is 2, and *b*_0_ is 1, formula (18) can be obtained, and the discrete wavelet can be expressed as

(20) $$\begin{array}{c} f\left(e\right)=I\overset{+\partial }{\underset{-\partial }{\sum }}\overset{+\partial }{\underset{-\partial }{\sum }}I_{m,n}\psi_{m,n}\left(e\right), \end{array}$$

(21) $$\begin{array}{c} f\left(e\right)=\int_{n}^{m}{\left(a,b\right)}^{-1/m-1}\partial \frac{1}{a-b}. \end{array}$$

Discrete approximation signal processing by high-pass filter is [22]

(22) $$\begin{array}{c} h_{i+1}l=h_{j}l\overset{L}{\underset{i=1}{\sum }}\left(\eta \pm \left(m,n\right)\right), \end{array}$$

(23) $$\begin{array}{c} h_{i+1,k}=\int_{a+1}^{2}\psi_{i+1,k}•\underset{k}{\sum }h_{j,k}. \end{array}$$

Combining the above two formulas can simulate the detailed rules of the high-frequency motion of the atomized particles to construct a model, assuming that it is represented by S, H in the decomposition process:

(24) $$\begin{array}{c} S_{m,n}=\underset{i}{\sum }g_{i-2n}w_{i+1,m}, \end{array}$$

(25) $$\begin{array}{c} H_{m,n}=\underset{i}{\sum }g_{2m-n}w_{m+i,n}. \end{array}$$

Atomized particles quickly recompose to a decomposed state [23]:

(26) $$\begin{array}{c} S_{m+1,n}=\underset{i}{\sum }\left(g_{i-2m}a_{m,n}+h_{i+2n}b_{i,m}\right). \end{array}$$

Equations *a* and *b*, respectively, represent the high-pass and low-pass parts of the atomized particle wave during decomposition and reconstruction [24].

## 3. Experimental Research and Data Analysis

### 3.1. Experiment Inclusion Criteria

1. Combined basic diseases, such as bronchopulmonary dysplasia, coronary heart disease with hemodynamic changes, incomplete delivery, low birth weight, neuromuscular disease, and cystic fibrosis
2. Assess whether there are high-risk factors for severe bronchiolitis, such as less than 12 weeks, premature delivery, and coronary heart disease with hemodynamic changes bronchopulmonary dysplasia
3. *Experimental Subjects*. Perform basic physical examination and medical history investigation of patients to form a clinical diagnosis of bronchiolitis and its severity. The age of the included clinical cases is concentrated in infants from 1 month to 9 months, with an average age of 1 month. In 2 to 6, there are 30 people in this experiment. 10 people are in the control group, 10 people in the experimental group A, and 10 people in the experimental group B

### 3.2. Experimental Process

1. Construct a model for the pathogenesis of bronchiolitis
2. Make statistics on the basic information of the hospital's entered cases in the past 8 years
3. To identify the 30 patients in this trial and evaluate the outcome of their pediatric capillary bronchitis treated with hypertonic saline nebulization therapy using a picture enhancement technique

- Observation group and outpatient physical examination infants and young children collected venous blood to obtain the consent of their families in advance. Children in the observation group were given intravenous infusion within 24 hours after hospitalization and one week after treatment in the morning. The normal group collected 2.0-2.5 ml of fasting peripheral venous blood in the early morning during the physical examination of the children's health clinic
- *3% Hypertonic Saline Nebulizer Inhalation*. Nebulizer inhalation of hypertonic saline is advisable for hospitalized children, but not for outpatients. The pathophysiological characteristics of bronchiolitis are airway inflammation and increased mucus secretion, so it is beneficial to increase the rate of cilia clearance

### 3.3. Experimental Analysis

The pathogenesis of bronchiolitis is still unclear. Most scholars believe that immune imbalance is an important factor affecting its pathogenesis and condition. Weakened humoral and innate immune functions will reduce the body's ability to resist infection, and pulmonary dysplasia is also considered to be bronchiolitis. Bronchiolitis is the most common lower respiratory tract disease in children and adolescents, especially affecting the health of children, and some children are susceptible to asthma. Reported studies have also proved that the prevalence of asthma in children with bronchiolitis is closely related to atopic physique. Children with atopic rules are prone to develop asthma after suffering from bronchiolitis, and a large number of scientists have also confirmed that the prevalence of asthma in children with bronchiolitis is higher than that in humans. The main disease that causes bronchiolitis is RSV, which can account for 75% during epidemics. Its RNA is wrapped in a shell containing 10 different glycoproteins, of which the combination of facial (F) glycoprotein and attachment (G) glycoprotein is the most important for virus production. We do not understand the pathogenesis of bronchiolitis, and we only build a model diagram based on our understanding, as shown in Figure 2.

The virus can cause direct damage to the respiratory tract. After infection, bronchiole epithelial cells appear necrosis, submucosal replacement, edema, gland hyperplasia, and increased mucus secretion, which can easily lead to stenosis and obstruction of the lumen, increased oxygen supply, and can cause emphysema and atelectasis. Inflammation can also spread to the alveoli, alveolar walls, and lung interstitium, causing inflammation and airway obstruction. In this experiment, 30 children from a hospital were selected for the study of hypertonic saline aerosolization treatment with image enhancement technology. By inhaling nebulized hypertonic saline, it acts on the respiratory tract to improve edema in the respiratory tract by means of decreasing osmotic pressure, accelerating clearance, and allowing secretions to be discharged as quickly as possible. First, relevant investigation preparations were carried out, and the number of pediatric bronchiolitis cases in the hospital in the past 8 years was counted, as shown in Figure 3.

Pulmonary function examination and clinical research in the history of more than 300 years, from the first liquid seal to the size of the tail to the lungs, and finally gradually developed to the commonly used electronic computer cooperation, the principle is to use the human respiratory physiology knowledge, plus modern medicine. The method in the examination understands and evaluates the functional status of the human respiratory system and can also calculate the therapeutic effects of respiratory diseases or chest diseases and pulmonary dysfunction, evaluate the safety of surgery, and predict postoperative respiratory function, etc., which can more objectively evaluate the lungs. The degree of functional impairment is also an indispensable method in the follow-up process in the future. The basic situation of the cases in the hospital was understood, and the data were recorded in Table 1.

As shown in Figure 3, patients with pediatric capillary bronchitis received at the hospital over an 8-year period showed an extremely rapid increase over time, with the highest number of years mostly concentrated in the last few years. As shown in Table 1, the clinical symptoms of the pediatric patients admitted to the hospital were mostly dyspnea, followed by coughing up blood.

According to incomplete statistics, the incidence of bronchitis varies in different periods: spring incidence is 12.28%, summer incidence is 33.58%, autumn incidence is 32.14%, and winter incidence is 8.47%. Differences were considered significant except between spring and autumn, when they were politically significant. How to decrease the duration of the illness and promptly minimize the signs and conditions is the primary study direction for therapy. The basic situation of these 30 experimental participants was understood, as shown in Figure 4, and Table 2 is the basic situation of the general information of these patients.

Bronchiolitis has a certain degree of its own primary support and treatment, but severe bronchiolitis in young infants can also cause serious adverse consequences. Antiviral drugs and aerosol inhalation of salbutamol and budesonide are generally effective. Early prevention should be an important means to reduce bronchiolitis infection. In order to provide targeted treatment to these patients, we classify and analyze the severity of their illnesses, as shown in Figure 5.

The physiology and anatomy of the human head are closely related. Compared with adult patients, due to the relatively narrow trachea and bronchi and the imperfect development of the surrounding elastic fibers, the airway resistance around infants and young children will account for a higher proportion of the total airway resistance. As a result, when the mucosa of the airway is infected, congestion and edema appeared, which can easily lead to narrowing of the airway. In addition, too much mucus cell secretion is not easy to pass out of the body, and it is more prone to blockage; in particular, infants and young children have incompletely developed vasculature in the fine-bronchial wall, the mucus cilia function is relatively poor, it is not easy to digest the excretion, and the blockage of airway will be more remarkable. Therefore, in infants with bronchiolitis, smooth muscle spasm causes less breathing, mainly due to eating and edema of the respiratory mucosa, obstruction of secretions, and obstruction of the respiratory tract. In this regard, it is necessary to choose atomization therapy to care for young children, and the simplified operation process is shown in Figure 6.

It is difficult for children to take medicine due to their special physical characteristics and physical factors. The technique of hypertonic saline nebulization therapy based on image enhancement is very sensitive, accurate, and less influenced by water vapor and has a wide linear range. In addition, this technique is a noncontact technique, which allows better avoidance of cross-contamination between patients, and works as shown in Figure 6.

At present, the common ones are compression atomizer, ultrasonic atomizer, mesh atomizer, etc.. We evaluate their performance levels (1-10), and the statistics are shown in Figure 7.

According to the data in the above figure, we can find that the treatment time of nebulization therapy is short, the amount of inhaled lung medicine is high, and large doses can be given multiple times. It has the advantages of large aerosol volume, low power, easy operation, and quietness and noise. The image enhancement technology is applied to the ultrasonic nebulizer and the net-type nebulizer before and after the three types of performance tests for the continuous administration of large doses, and the amount of aerosol and the amount of inhaled lung drugs are tested. The results are shown in Figure 8.

To better guide the clinical application of this pulmonary function testing technology, there are strict performance rules for pulmonary resuscitation and spirometry, as well as enhanced quality control related to tidal breathing and pulmonary function testing. Signal analysis provides insight into changes in airway function. The impact of data analysis atomization processing on the application of imaging techniques is shown in Figure 9.

The evaluation of the above data mainly focused on the acute phase (cough, wheezing, shortness of breath, wheezing, and scattered or diffuse wheezing or rales in the lungs) of the bronchiolitis group at admission and the remission phase before discharge. Through a comparative analysis with the comparison group, a tidal lung function test was performed 3 and 6 months after discharge to compare the differences in various parameters of the lung function. The data was also recorded during the observation period, as shown in Figure 10.

The gastrointestinal severity of the main symptoms and signs on the third day after treatment was compared between the two groups. There was no difference in the progression speed of asthma, sputum, fever, and pulmonary symptoms. Compared with the reduction rate of asthma score, the asthma symptom reduction rate of the treatment group on the 3rd day after treatment was greater than that of the control group; it was greater than that of the control group, indicating that the treatment group was better than the control group on the 7th day after treatment. In this regard, corresponding scoring statistics are carried out, as shown in Table 3.

X-rays of bronchiolitis showed patchy infiltration shadows around the bronchi, emphysema, hyperinflation, and other phenomena, as well as local atelectasis. Eosinophilic inflammation dominates in the later stage of bronchiolitis, indicating that bronchiolitis should be a mixed airway inflammation of eosinophils and neutrophils. The physical and chemical properties of blood salt are closely related, and antimicrobial therapy is well tolerated and safe for children. In terms of onset time, image-enhanced nebulization therapy improves symptoms such as cough and asthma in children with bronchiolitis and is more effective than drug therapy alone. The effect is shown in Figure 11.

Bronchiolitis is often associated with multiple organ system damage, and the effects of complications vary. It can affect the heart, gastrointestinal tract, brain, etc. Among them, the most common damage to the digestive system is heart damage. The deterioration of the digestive system is manifested as diarrhea, occasional vomiting, constipation, etc. Heart injury is commonly manifested as elevated myocardial enzyme spectrum and abnormal electrocardiogram, etc. Heart failure may occur in severely ill children. According to this phenomenon, each function of the test group was checked, as shown in Table 4.

Comparison before and after self-treatment: after treatment, the total number of symptoms and signs of the treatment group and the control group was significantly reduced compared with that before the treatment. The difference was statistically significant, indicating that the treatment group and the control group had more symptoms and signs and were more advanced than before the treatment. It is effective in improving the symptoms and signs of children with bronchiolitis.

## 4. Discussion

Aerosol inhalation of blood salt can increase the local osmotic pressure of the airway, which can not only dissolve the exhalation and make saliva easier to discharge but also promote water absorption in the submucosa of edema and edema, thereby reducing respiratory mucosa and edema interstitial. Carry out important nursing measures for children, such as sputum expectoration and low back pain during inhalation treatment, close monitoring of behavior after taking the medicine, timely treatment of adverse reactions, and health education for the children's family members. Data show that after hypertonic saline treatment in children with bronchiolitis, the hospital stay, the time to relieve wheezing symptoms, the time to reduce cough symptoms, and the time to improve lung signs are all reduced, and there is no way to find it serious side effects. The treatment group's tremor, cough, lung murmur elimination time, and hospitalization time were shorter than those of the control group, and the effective rate was improved, indicating that both affect the consistency of bronchiolitis treatment, and the combination of the two has the best effect in the control group and symptoms. Significant differences existed in the elimination time of signs and the number of days in hospital. In addition, the use of interferon and hypertonic inhalers is easy to operate and will not produce adverse reactions during the treatment process, which reduces a lot of auxiliary treatment funds in the treatment of bronchiolitis.

## 5. Conclusion

For individual infants and young children, bronchiolitis has the characteristics of multiple attacks. If the infant is genetically prone to allergies, then, it is likely to have repeated persistent wheezing. This process is typical asthma symptoms. In this regard, allergic physique is an important factor that promotes the aggravation of bronchiolitis. Indoor and outdoor factors, especially environmental factors such as air pollution, can cause chronic inflammation of the airways and cause repeated wheezing. The recent rapid increase in respiratory tract viral infections, influenza, parainfluenza, rhinovirus, adenovirus, and other cases of mycoplasma infection is also another important factor in causing bronchiolitis, causing lethargy; reducing the incidence of childhood asthma may reduce the incidence of childhood asthma rate. Considering that it may be related to the different physiological characteristics of different age groups, that is to say, the poor immunity of children under 1 year old causes the spread of pneumonia bacteria to easily spread to the entire lung; and the older children who are compared with this have various physical functions. The response gradually matures, and the energy to resist infection continues to increase. Younger, low-weight children have poor resistance to diseases and stimuli and are prone to complications and harmful consequences. Therefore, the operator needs to have a superb technical level and be good at dealing with problems in this field. It is groundbreaking to transform the raw image informations into a more adequate human-machine discrimination methodology and to use the messages available from those images of medicine for the image knowledge of the condition of the children with bronchiectasis and for the mediation of the nebulization treatment data. This method can relieve bronchospasm to a large extent, reduce the adverse reactions caused by airway inflammation, and reduce airway hyperresponsiveness, thereby reducing the number of attacks and reducing the degree of wheezing, so as to effectively control wheezing, the purpose of improving lung function.

## Figures and Tables

**Figure 1:** Comparison chart of image enhancement processing.

**Figure 2:** Pathogenesis of bronchiolitis.

**Figure 3:** The number of cases of pediatric bronchiolitis in the past 8 years.

**Figure 4:** The basic picture before treatment.

**Figure 5:** 30 severity of bronchiolitis in children before treatment.

**Figure 6:** Nebulization therapy for bronchiolitis in children.

**Figure 7:** The performance of different aerosol therapy machines.

**Figure 8:** Image enhancement technology and nebulization treatment.

**Figure 9:** Treatment effect statistics of the three groups of children.

**Figure 10:** Data record of efficacy observation after treatment.

**Figure 11:** The effect of image enhancement nebulization treatment.

**Table 1:** Clinical characteristics of patients with bronchitis.

Clinical features	Number of cases	Composition ratio
Difficulty breathing	56	32.1%
Cough	38	27.9%
Hemoptysis	44	29.5%
Hoarse	13	8.3%

**Table 2:** General data sheet of the patients participating in the experiment.

Group	Gender		Age (month)	Course of disease
	Male	Female		
Control group	5	5	4.21 ± 1.23	4.11 ± 1.21
Experimental group A	3	7	3.27 ± 1.49	3.44 ± 1.45
Experimental group B	7	3	5.27 ± 1.08	5.43 ± 1.11

**Table 3:** Tal scoring criteria after treatment.

Respiratory rate		Wheeze	Blood oxygen saturation
<3 months	≥3 months	Not	≥90%
31-45	41-55	Weak	90-94%
46-60	56-70	Weak	80-89%
>50	>60	Not	<80%

**Table 4:** Comparison of total effective rates of the three groups (*m*).

Group	*m*	Effective	Invalid	Markedly effective	Total effective
Experimental group A	10	8	0	8	27.6%
Experimental group B	10	9	0	7	23.3%
Control group	10	5	2	3	10%

## Data Availability

We do not have permission to share data from the data provider.
